The article "Face detection based on K-medoids clustering and associated with convolutional neural networks" was retracted in 2025. Reasons: suspected computer-generated content; unreliable results or conclusions; concerns about the citations.

# Face detection based on K-medoids clustering and associated with convolutional neural networks

**DOI:** 10.1016/j.heliyon.2024.e35928

**Published:** 2024-08-08

**Authors:** Potharla Ramadevi, Raja Das

**Affiliations:** Department of Mathematics, School of Advanced Sciences, Vellore Institute of Technology (VIT), Vellore, 632014, Tamil Nadu, India

**Keywords:** K-medoid clustering, Convolutional neural networks, K-means clustering, Fuzzy K-Means clustering, SVM, DenseNet201

## Abstract

Over the last several years, the COVID-19 epidemic has spread over the globe. People have become used to the novel standard, which involves working from home, chatting online, and keeping oneself clean, to stop the spread of COVID-19. Due to this, many public spaces make an effort to make sure that their visitors wear proper face masks and maintain a safe distance from one another. It is impossible for monitoring workers to ensure that everyone is wearing a face mask; automated solutions are a far better option for face mask identification and monitoring to assist control public conduct and reduce the COVID-19 epidemic. The motivation for developing this technology was the need to identify those individuals who uncover their faces. Most of the previously published research publications focused on various methodologies. This study built new methods namely K-medoids, K-means, and Fuzzy K-Means(FKM) to use image pre-processing to get the better quality of the face and reduce the noise data. In addition, this study investigates various machine learning models Convolutional neural networks (CNN) with pre-trained (DenseNet201, VGG-16, and VGG-19) models, and Support Vector Machine (SVM) for the detection of face masks. The experimental results of the proposed method K-medoids with pre-trained model DenseNet201 achieved the 97.7 % accuracy best results for face mask identification. Our research results indicate that the segmentation of images may improve the identification of accuracy. More importantly, the face mask identification tool is more beneficial when it can identify the face mask in a side-on approach.

**Table:** Abbreviation

CNN	Convolutional Neural Networks
DCNN	Deep Convolutional Neural Networks
SVM	Support Vector Machine
FKM	Fuzzy K-Mean Clustering
WHO	World Health Organization
AI	Artificial Intelligence
ML	Machine Learning
CCTV	Closed Circuit Television
CBIR	Content-Based Image Retrieval
PAM	Partitioning Around Medoids
CLARA	Clustering Large Applications
ROC	Receiver Operating Characteristic
AUC	Area Under the Curve
TP	True Positive
TN	True Negative
FP	False Positive
FN	False Negative
TPR	True Positive Rate
FPR	False Positive Rate

## 1 Introduction

Face mask detection has several uses in real-world situations, including remote surveillance of individuals and real-time biometrics. Criminals often cover their faces around the mouth. Researchers have already found a solution to the challenge of detecting occluded faces in the form of a person's head and shoulders [1]. The need to constantly verify many people for using face masks makes this work more difficult. Additionally, the new coronavirus illness (COVID-2019) outbreak required the use of face masks and various additional limitations. The World Health Organization (WHO) declared COVID-19 a pandemic and suggested many preventative measures [2], including the use of face masks, because of their deadly effects, quickly spread, and lack of proper medication and medical care [3,4]. In certain nations, wearing a face mask is required for admission into public buildings. However, the manual inspection process is impossible since so many people use government buildings, and public spaces like airports railway stations, and retail centers. The study of face mask's automated identification and detection has recently attracted interest. Researchers have begun developing automated detection systems to assist with monitoring and surveillance applications during COVID-19 [5]. Identification and classification are two tasks involved in the detection of face masks since it is necessary to identify faces to determine whether people are wearing masks. The research group created Many face-detection approaches, making the first task a heavily researched issue in computer vision [6]. The identification of face masks on various datasets has been the subject of a lot of effort in the last year [7].

The article "Face detection based on K-medoids clustering and associated with convolutional neural networks" was retracted in 2025. Reasons: suspected computer-generated content; unreliable results or conclusions; concerns about the citations.

Before declaring using a mask is the most effective way to stop the coronavirus from spreading, getting the government and other authorities to enforce mask wear in public spaces can be difficult. At least artificial intelligence (AI) applications that use machine learning (ML) or deep learning algorithms (DL) may detect masks in real-time utilizing a built-in surveillance add network (network of CCTV cameras or any other) that may help in forcing the wearing of masks in open spaces. It is a simple method of maintaining social quiet, having people under control locally, and ensuring that everyone is wearing masks [8]. The technique of recognizing pixels that belong to the same region and assigning them a common name is the fundamental aspect of picture segmentation. Therefore, a wide range of industries, including object identification [9], moving object tracking, and medical image processing [10], have widely used image segmentation. For the first time, this paper uses image segmentation for face mask detection to get high accuracy.

The article "Face detection based on K-medoids clustering and associated with convolutional neural networks" was retracted in 2025. Reasons: suspected computer-generated content; unreliable results or conclusions; concerns about the citations.

The foundation of picture recognition and comprehension is image segmentation [11]. The method of classifying data items into several groups or classes is known as clustering [12]. Image segmentation commonly uses K-means, a traditional technique for grouping analysis difficulties. The original cluster centers have a significant impact on the K-means clustering process. distinct clustering outcomes might arise from distinct starting cluster centers. In the K-means algorithm, you need to specify an initial number of clusters (K) which are randomly chosen at the beginning. That means it is frequently challenging to identify the optimal K value with accuracy.

The K-medoid clustering approach represents the center, or medoid, of a cluster as an actual location within the cluster. The heart of a cluster is home-based to the medoid, or cluster center [13]. The location of the medoid is also the spot where the total distances to all other objects are the lowest. Because of its resilience to noise and outliers, a medoid can serve as an accurate cluster center representation. In this technique, start with K objects (points) and iteratively work our way up to the best cluster objects (points). Next, our work examined every possible combination of points and determined the quality of clustering for each pair of points. The preset work is to replace the existing best object with a new object (point) if the located one with the best-improved distortion function value.

The primary reason for the industrial relevance of K-medoid clustering for face classification is its effective processing of large data sets. When compared to other clustering methods like FKM. K-medoid clustering is more resilient to outliers. This resilience is useful for accurately grouping facial characteristics in face classification, where the existence of outliers (for example, significant lighting conditions and occlusions) is commonplace. K-medoid clustering helps classify faces by giving each cluster a medoid that represents common facial features. It is appropriate for face classification jobs since it is robust and capable of handling huge datasets with ease. K-medoid clustering enables the inclusion of information such as pixel intensities and face landmarks by providing flexibility in the definition of the distance metric. Its characteristics enable it to adjust to various jobs and situations. K-medoid clustering yields clusters that are useful for Content-Based Image Retrieval (CBIR) and image retrieval, which makes it crucial for industrial applications such as picture databases and security systems.

There is limited research and data on face mask detection [14]. Most entries regarding mask usage are concise and simply indicate whether masks are present. In the field of computer vision, researchers have advanced various cutting-edge techniques, especially in deep learning, for object detection, recognition, tracking, and scene understanding. These advanced methods offer effective solutions for face mask detection by identifying visual entities or objects within images that belong to specific categories. Consequently, deep learning-based models for detecting and identifying face masks have become a crucial computer vision task, supporting healthcare systems and the global community [15]. Techniques such as CNNs can be employed to create intelligent surveillance systems that detect mask-wearing individuals and evaluate social distancing in public spaces [16].

The article "Face detection based on K-medoids clustering and associated with convolutional neural networks" was retracted in 2025. Reasons: suspected computer-generated content; unreliable results or conclusions; concerns about the citations.

The convolutional properties of the DCNN (Deep Convolutional Neural Network) using VGG19 with a spatial attention method. The method is designed for accurately classifying traffic incidents with an average accuracy of 93.72 % [17]. DenseNet201 [18] is an existing iteration based on the dense-network concept, this design uses a unique method that connects each layer feed-forward to every other layer. In addition, the DenseNet201 model integrates a blend of pooling layers and a compact structure. As a consequence, these design decisions help to decrease the number of parameters and the overall complexity of the model, leading to enhanced efficiency.

Face recognition in computer vision is determining a person from their face image. The well-known CNN model VGG16 (Simonyan and Zisserman, 2015) [19] has been trained on various image datasets to improve its feature extraction skills and perform well in facial recognition applications. The face-detection approach is based on CNN pre-trained models and SVM. Due to its clear classification effect on nonlinear data, utilizing SVM [20] as our final classifier to recognize faces after feature extraction is complete. SVM offers several unique advantages regarding high-dimensional, nonlinear, and small-sample pattern recognition. SVM is also applicable to other machine learning issues including the curse of dimensionality and function overfitting. SVM is used in our system to do further feature extraction and ultimate classification using the face characteristics that are taken from CNN. In this method, we may potentially extract a greater number of characteristics than just CNN.

The novelty of this research paper is to create CNN with pre-trained models DenseNet201, VGG-16, and VGG-19 with SVM for classification that can identify who is wearing masks or not wearing masks. Before that, we used image segmentation to remove the noise data from the images. The proposed method is shown in Fig. 3. The model identifies people in the public setting who are not wearing masks by using the DenseNet201 model from the security cameras. Overall workflow as shown in Fig. 2.

The article "Face detection based on K-medoids clustering and associated with convolutional neural networks" was retracted in 2025. Reasons: suspected computer-generated content; unreliable results or conclusions; concerns about the citations.

In this contribution, datasets have been assessed by data-driven, unsupervised face detection methods from the literature review Table 1. Totally 2000 images were used from the dataset, which is utilized for clustering to lower the data noise and then K-medoids clustering to group the samples. The item that is most central within a group and has the least average distance from other entities is known as the medoid. The procedure identified as K-medoids aims to reduce the total differences between every data point and its nearest medoid. To lessen the K-medoids clustering algorithm's computing load, a hybrid strategy is suggested. The proposed model DenseNet201 can accurately identify face masks. For dependable face mask identification, our unique end-to-end DenseNet201 model automatically extracts the most discriminating characteristics. To assess the effectiveness of the face mask identification technique to create an extensive dataset. To demonstrate the effectiveness of our model, extensive tests were conducted to compare its performance with three pre-trained models using SVM for face mask classification.

**Table 1:** Summary of literature review.

Author	Face dataset	Method	Accuracy
Li, Yang, and Wu 2020 [37]	WIDER FACE Face dataset	Multi-Task Cascaded CNN with Inception-V2	96.35 %
Biju and Edison 2020 [38]	CEW database	Convolutional neural networks	80.9 %
Mellouk and Handouzi 2020 [39]	EMOTIC dataset	Convolutional neural Networks	86.4 %
Saravanan et al., 2022 [40]	Face image dataset	CNN with VGG 16	96.5 %
Agarwal, Itondia, and Mishra 2023 [41]	RMFD dataset	Extreme Learning Machine (ELM)	97 %
Balasubaramanian et al., 2023 [42]	Face mask dataset	Depth-wise Separable Convolutional Neural Network (DWSC-NN)	94.16 %
Dash, Sethy, and Behera 2023 [43]	Plant village dataset	CNN with DenseNet201	94 %
Rahman et al., 2023 [44]	FMPD real dataset	CNN with MobileNet	81.95 %

The following are the paper's main contributions.

• Developed a face dataset from different poses, and directions, with mask without mask images using a multiple free online database of face images.
• For face image segmentation, a new region-based clustering method known as K-medoid clustering has been proposed.
• To increase the identification accuracy of existing recognition techniques for face mask detection, convolutional neural network pre-trained models(VGG16, VGG19, and DenseNet201 were used.
• A comparative study of different methods for face mask dataset pre-processing and applied the pre-trained models to improve the accuracy.
• The proposed model DenseNet201 approach is evaluated using F1-score, precision, sensitivity, specificity, and accuracy.
• The development of an automated face mask detection system that enables real-time detection with little resource use. The rest of the sections of this paper are structured as follows: section 2 represents the related works. In section 3, the presented methodology. The method is explained in detail. Section 4 presents the results while section 5 presents the conclusion of the presented method.

The article "Face detection based on K-medoids clustering and associated with convolutional neural networks" was retracted in 2025. Reasons: suspected computer-generated content; unreliable results or conclusions; concerns about the citations.

## 2 Related work

There continues to be assurance for machine vision systems in the areas of computer vision, face, and skin recognition, etc. Applications for image processing have demonstrated that analyzing images is a successful technique for research. The identification of face masks is a crucial problem that requires the development of sophisticated automatic detection methods. The advancements in machine learning and deep learning have made it feasible to detect faces using technology rather than human observation.

Our objective is to create a more straightforward and effective K-medoid clustering technique. For the same goal, various other ways are accessible in the published works. Rather than applying PAM to all objects in a dataset. kambe, and Pe et al. [21] created CLARA, which applies PAM to derived objects only. CLARA's effectiveness deteriorated with the addition of more clusters, according to Verma et al. [22] suggested a method that maximizes the silhouette rather than minimizing the sum of distances to the nearest medoid. The suggested technique aims to balance network energy usage while extending its lifespan. To combine local search with the K-medoids algorithm and global search by the particle swarm optimization method [23], the hybrid K-medoids and QKSCO algorithm.

The dimension of the feature space is a common basis for splitting FKM approaches into two categories. The first speaks of executing fuzzy clustering in the initial high-dimensional space. Another method, known as extended FKM clustering, teaches the fuzzy membership connection in the low-dimensional space. All characteristics provide the same weights to the membership relationship learning for the first class of FKM algorithms. Numerous fuzzy theories and techniques have been developed recently to enhance the functionality of the original FKM [24]. To build a data entropy-based split network, for instance, maximum entropy fuzzy clustering techniques are given. These algorithms have a distinct physiological significance. With a weaker restriction on the membership, Pal et al. [25] suggested a possible FKM method that combines FKM and possibilistic K-Means. A few researchers additionally take into account the geometric details of a single pixel and the impact of the neighborhood to produce excellent picture segmentation results [26].

The article "Face detection based on K-medoids clustering and associated with convolutional neural networks" was retracted in 2025. Reasons: suspected computer-generated content; unreliable results or conclusions; concerns about the citations.

Abou Chaaya et al. [27]suggested a CNN model with two-stage neural networks for detecting face masks in crowded areas. Additionally, the researcher proposed a CFMD-Net which is a two-stage detector to overcome the crowded environment situation. The results showed that the average categorization accuracy was 96.5 %. Deep learning models, as opposed to shallow models, have recently become more popular in the development of object identification algorithms [28]. Because of this development, it is now believed that deep learning models are more capable of completing complicated tasks than shallow models. The creation of a model or system that works in real-time and can tell if people are wearing masks or not when used in public places would be a nice example of technology. Employed real-time deep learning to identify and differentiate emotions, using VGG-16 to classify seven faces [28]. This tactic works effectively during the current COVID-19 lockdown phase, which aims to halt the disease's future spread. Principal analysis of components was also used to distinguish between persons who had their faces covered from those whose have them uncovered [29].

In terms of datasets and detection methods, this section gives a broad overview of the literature on face mask detection. Several computer vision problems, including face identification, face tracking, face retrieval, and face occlusion detection have been the focused. Researchers used PCA [30], SVM [31], and Markov models [32] to carry out different tasks related to face occlusion detection, including head identification, facial feature detection, mask detection, skin color-based detection, and face parts detection. Low-resolution images of the monitoring instruments were the biggest problem for this research.

Shijie et al. [33]introduced a transfer learning method for the identification and categorization of pests and illnesses affecting tomato plants, using VGG16. Additionally, the experimented VGG16 feature extractor with SVM as a classifier with an average accuracy of 89 %. The VGG16 method to transfer learning outperformed the VGG16+ SVM strategy. Hemming et al. [34]have suggested a method that uses a deep CNN model to identify tomato whiteflies and the bugs that prey on them. The yellow sticky trap method was used to manually count the insects, and the results were compared. The results showed that the average categorization accuracy was 87.40 %. This research work finds the research gap in the literature review improves the high accuracy level using the K-medoid clustering for image segmentation.

The article "Face detection based on K-medoids clustering and associated with convolutional neural networks" was retracted in 2025. Reasons: suspected computer-generated content; unreliable results or conclusions; concerns about the citations.

Sheikh and Zafar et al. [35]suggest a transfer learning method MobileNetV2, ResNet50, and EfficientNet-B2, against such attacks, a face mask detection algorithm that is resilient to adversarial attacks with an accuracy of. For a similar scenario, the proposed transfer learning method with only a single fine-tuning MobileNetv2 achieved a better accuracy of 92.79 %. In both above works, researchers have experimented with the fast gradient sign method (FGSM) and projected gradient descent (PGD) for face mask detection [36].

## 3 Methodology

### 3.1 Data description

Fig. 1 incorporates both types of images owing to the absence of a standardized dataset for the detection of face masks and recognition of masked faces. The 2000 different types of images from the dataset utilized in this research, which includes data both with mask and without mask in different poses light condition images as shown in Fig. 1, were taken from the Kaggle repository [45]. Different datasets are needed for each of these activities. Facemask detection makes up the bulk of our datasets. Only 2000 images from the dataset were taken into consideration. The face mask detection images collection consists of photographs of faces with and without masks as shown in Fig. 1. Because square-shaped images (usually 224 × 224 × 3 pixels) are often used as inputs by traditional AI deep models, additionally total pixels to the boundary of several images. Finally, each picture was cropped and resized to 224 × 224 × 3 pixels using bilinear interpolation.

**Fig. 1:** (a–b) Represents the sample images of our dataset.

**Fig. 2:** Block Diagram of the overall work system.

**Fig. 3:** Demonstrate Block diagram of the proposed method.

### 3.2 Image segmentation for using the clustering methods

#### 3.2.1 K-means clustering

This method is particularly useful in image processing, where it can segment images into distinct regions based on pixel similarities, enhancing the ability to detect and analyze specific features. By reducing the complexity of the data and highlighting important structures, K-means clustering aids in improving the accuracy and efficiency of machine learning models. The K-means cluster analysis is the partitioning technique used most often.

This is how the algorithm works.

(1) Choose K centroids (K randomly selected rows).
(2) Pick K items at random from the data collection to serve as the first cluster means or centers.
(3) Based on the Euclidean distance between the item and the centroid, assign each data point to its nearest centroid.
(4) The new mean values of each of the K cluster's data points are calculated to update each cluster's centroid.

The article "Face detection based on K-medoids clustering and associated with convolutional neural networks" was retracted in 2025. Reasons: suspected computer-generated content; unreliable results or conclusions; concerns about the citations.

A vector of length p that contains the K-means of all the variables for the observations in the cluster is the centroid of a $k^{th}$ cluster; p is the number of variables.

Repeat steps 3 and 4 until the cluster assignments stop shifting or you reach the optimum number of repeats.

$X=\left[x_{1},\ldots ‥x_{n}\right]\in R^{d\times n}$ where d is the number of features and n is the number of data points. Finding the data split that minimizes the following eq. (1) objective function is the goal of the K-means clustering technique.

(1) $$J\left(X,V\right)=\sum_{j=1}^{k}\sum_{x_{i}\in X_{j}}\|x_{i}-v_{j}|{|}_{2}^{2}\text{,}$$

Where K is the number of clusters, $v_{j}$ is the cluster center of the $j^{th}$ cluster, and contains data points that belong to the $j^{th}$ cluster.

It $H=\left\{h_{ij}\right\}\in R^{n\times k}$ is the cluster indicator matrix and its element is defined as $h_{ij}=1$ if it belongs to the $j^{th}$ cluster, and otherwise. Then, the objective function of K-means can also be written as following eq. 2

(2) $$\min_{H,V}\sum_{i=1}^{n}\sum_{j=1}^{k}h_{ij}\|x_{i}-v_{ij}|{|}_{2}^{2}\text{.}$$

Iteratively minimizing the sum of distances between each element and its cluster centroid for K clusters is the foundation of the K-means algorithm. As soon as the total cannot be dropped anymore, the samples are moved across clusters.

#### 3.2.2 Proposed method K-medoids

The K-medoid clustering algorithm employs a medoid or actual cluster point to serve as the representative center of the cluster. The center of a cluster is typically identified by a method or a cluster center, as noted in sources [46].

Furthermore, the medoid is situated at the minimum total distance from all other entities (points). The utilization of a medoid as a cluster center is deemed effective in accurately representing the cluster center, primarily due to its robustness against noise and outliers. The PAM algorithm is a widely used K-medoid clustering technique. The algorithm initiates by selecting K objects or points and subsequently iteratively approaches the optimal cluster objects or points. Subsequently, the clustering efficacy is evaluated by scrutinizing all possible point pairings. If an object (point) is identified with the most optimal distortion function value, it shall supersede the present best object (point). The recently produced optimal entities, referred to as points, comprise the upgraded and refined medoids. The algorithm aims to minimize the disparity between objects and their corresponding reference points. The process assists in reducing the total amount of differences between a given entity and its nearest neighboring cluster. To clarify, the K-medoids algorithm endeavors to minimize the objective function known as the absolute error (E). The aforementioned function is presented in the form of an eq. (3).

(3) $$\text{Absolute}\;\text{error}\left(E\right)=\sum_{j=0}^{k}\sum_{p\in c_{j}}^{n}\left|p-ob_{j}\right|$$

In the context of cluster analysis, Eq. (3) the sum of absolute error (E) is denoted as a function of a data point (p) that represents an object within the cluster. Additionally, the representative object of the cluster $\left(C_{j}\right)$ is also denoted. The above-mentioned procedure is repeated until the object within the cluster that is $\left(C_{j}\right)$ situated at the centremost position, also known as the medoid, is attained. The present study involves the development of the K-medoids algorithm to cluster n objects into k clusters.

The article "Face detection based on K-medoids clustering and associated with convolutional neural networks" was retracted in 2025. Reasons: suspected computer-generated content; unreliable results or conclusions; concerns about the citations.

The grayscale image is segmented using a K-Medoids clustering-based technique to separate the facial region from the background. The results show that the K-Medoids are more resilient to noise and outliers when compared to K-means and FKM [47]. The K-Medoids technique selects one real data point from that dataset to be used as each cluster center, in contrast to the K-means approach, which utilizes the average of connected data points in the provided dataset to represent the cluster centers. Fig. 3 displays the block schematic for the segmentation procedure. Using the K-Medoids clustering approach, the K value indicates the number of clusters that need to develop. The K-Medoids clustering technique is used to segment the face region after initializing K = 4 and receiving the grayscale face picture with a mask and without a mask. Therefore, the face image is reduced from the surrounding region on the face mask surface image. Fig. 11 displays the result of grouping facial images using K-medoids.

#### 3.2.3 Fuzzy K-Means clustering

This method is used for the pre-processing of the images it will work the segment the face mask images. FKM assigns each data point to a single cluster with full membership (0 or 1) and allows partial membership. Each data point belongs to all clusters with varying degrees of membership represented by values between 0 and 1. This method is one of the original algorithms projected to manage overlap clusters [24]. FKM is predicated on assigning each data point to numerous cluster samples based on its degree of participation. Technically, a data set is represented $X=\left[x_{1},\ldots ‥x_{n}\right]\in R^{d\times n}$ where n is the number of data points and d is the dimension. $x_{i}\in R^{d}$ is the point of data. Assume that these data points correspond to c clusters. The objective of FKM is to divide n data points into C clusters in the absence of label information [48] is defined as following Eq. (4).

(4) $$\min_{U,M}\sum_{i=1}^{n}\sum_{k=1}^{c}u_{ik}^{h}\|x_{i}-m_{k}|{|}_{2}^{2}\text{,}$$

$$s.t\sum_{k=1}^{c}u_{ik}=1,0\leq u_{ik}\leq 1\text{,}$$

The fuzzy exponent h, which is often modified to a real value greater than 1, is used for modifying the fuzzy degree. $u_{ik}$ is the component of the matrix $U\in R^{n\times c}$ and represents the amount of the $i^{th}$ data points membership in the cluster. $m_{k}$ is the prototype cluster for the $k^{th}$ cluster, and $M=\left[m_{1},\ldots ‥m_{c}\right]$. By modifying the parts of U and M according to the following Eq. (5) and Eq. (6) instructions may get the best resolution to problem (1):

(5) $$u_{ik}=\frac{1}{\sum_{k=1}^{c}{\left(\frac{{\left\|x_{i}-m_{k}\right\|}_{2}}{{\left\|x_{i}-m\right\|}_{2}}\right)}^{\frac{2}{h-1}}}\text{,}$$

And

(6) $$m_{k}=\frac{\sum_{i=1}^{n}u_{ik}^{h}x_{i}}{\sum_{i=1}^{n}u_{ik}^{h}}\text{.}$$

When h = 1 the problem (1) is equal to

$$\min_{U,M}\sum_{i=1}^{n}\sum_{k=1}^{c}u_{ik}\|x_{i}-m_{k}|{|}_{2}^{2}\text{,}$$

$$s.t\;\sum_{k=1}^{c}u_{ik}=1,u_{ij}\in \left\{0,1\right\}\text{,}$$

It is precisely the intended purpose of k-means. If the first cluster examples are provided, U is calculated as.

The article "Face detection based on K-medoids clustering and associated with convolutional neural networks" was retracted in 2025. Reasons: suspected computer-generated content; unreliable results or conclusions; concerns about the citations.

### 3.3 Convolutional neural networks approaches

The image-take technique creates a facial picture collection that includes every surface problem. Preprocessing involved K-medoid, K-means, and FKM clustering to eliminate noise from the obtained picture. Following the application of the filter, facial surface pictures are separated from the background area using clustering methods. The CNN received the dataset's separation image through segmentation for training. Utilized the three distinct CNN models VGG 16, VGG19, and DenseNet201 with SVM for face classification.

CNNs are an important tool in machine learning. The whole CNN algorithm structure consists of an input layer, convolutional layers, pooling layers, fully connected layers, a classification layer, and at last the final output layer [49]. Fig. 4 illustrates the CNN's internal structure. The essential element of CNN is the convolutional layer. It performs a process known as a “convolution operation” which uses a filtering technique to build an activation on an input. It is possible to extract features from a picture, such as edges, textures, and objects, by employing convolutional layers. Updates to the filter weights during training led to the creation of the feature maps. Max-pooling and average-pooling are the two types of pooling layers, and both are used to reduce the top layer's dimension. The combination of the convolution and pooling layers qualifies it as a feature extractor. The completely linked layers are used during the classification step [50]. ReLU (Rectified Linear Unit) is a popular activation function in CNNs because of its straightforward implementation and high performance. Represented as ReLU(x)=max(0,x) Where x is the input to the neuron. This function outputs x if x is positive; otherwise, it outputs 0. It provides non-linearity, computational efficiency, and sparse activation by passing through positive inputs unchanged while outputting zero for negative inputs. This property helps to alleviate the vanishing gradient problem, enabling quicker and more consistent convergence during the training process.

The article "Face detection based on K-medoids clustering and associated with convolutional neural networks" was retracted in 2025. Reasons: suspected computer-generated content; unreliable results or conclusions; concerns about the citations.

**Fig. 4:** Architecture of convolutional neural networks.

The SoftMax function is used to convert features into class probabilities. This layer includes the same number of units as classes. The SoftMax function is given by Eq. (7).

(7) $$Soft\;\max\left(a_{i}\right)=\frac{e^{a_{i}}}{\sum_{j=1}^{m}e^{a_{j}}}$$

Where SoftMax ($a_{i})$ and $a_{i}$ represent the probability and feature of the class, respectively. The denominator is used to regularize the probability distribution across *m* classes.

The learning rate (α) is an essential hyperparameter in CNNs that determines the step size for updating the network's weights during training. It specifies the magnitude of adjustments made to the model in response to the calculated error with each weight update. Table 2 shows the CNN hyperparameters used with different pre-trained models throughout the training process.

**Table 2:** Face mask detection of CNN pre-trained models Hyperparameters.

Parameters	VGG 16	VGG19	DenseNet201
**Learning Rate**	0.01	0.01	0.001
**Batch size**	32	32	32
**Epochs**	30	30	30
**Input layer size**	224 × 224× 3	224 × 224× 3	224 × 224× 3

Face verification has made major advancements as a result of CNN's recent success. our suggested CNN-based models VGG-16, VGG-19, and DenseNet201, in this area. This research concentrated on the network architecture of the proposed CNN since the structure of CNN has been described in several studies [51].

The suggested simulation uses VGG-16, VGG-19, and DenseNet201, three distinct pre-trained DCNN models. The images have been downsized to a standard size of 224 × 224 pixels to match the default input size of the VGG-16, VGG-19, and DenseNet201, CNN architectures as shown in Fig. 5, Fig. 6. This is a result of the various image sizes in the extended face image collection of data. Throughout the training process, utilized the image objects to help reduce over-fitting, a common issue when using pre-trained CNN models with limited data.

The article "Face detection based on K-medoids clustering and associated with convolutional neural networks" was retracted in 2025. Reasons: suspected computer-generated content; unreliable results or conclusions; concerns about the citations.

**Fig. 5:** (a–b) Represents the architecture of CNN pre-trained models.

**Fig. 6:** Architecture of DenseNet201.

#### 3.3.1 VGG-16 and VGG-19

The first layer of the VGG-16 and VGG-19 network in the proposed models, as illustrated in Fig. 5 has been supplied with the 224 × 224 pixel images for feature extraction [52]. VGG-19 and VGG-16 are two different ⁠ designs of the VGG network. The number of layers in each design is represented by the numbers 16 and 19. For example, VGG-16 has 16 convolutional layers, 3 fully connected layers, 5 max-pooling layers, and 1 SoftMax layer. 13 convolutional layers, two fully linked layers, and one SoftMax classifier make up this structure. The image processing begins with ⁠ multiple convolutional layers. A 224 × 224-pixel image goes through the first set of two convolutions ⁠ with a receptive area of 3 × 3 after applying ReLU activation functions. Each level has ⁠ 64 filters. The stride value is always set to 1, and padding ⁠ remains at one pixel to maintain full spatial resolution. Thus, the output activation dimensions match ⁠ those of the source images. ‍Next, the activations are sent to a pooling layer with a stride value ⁠ of 2 pixels since the window size is set to 2 × 2. This reduces the magnitude of ⁠ activations by half. At this point in the first stack, ⁠ the output size becomes 112 × 112 × 128.

The output from this stage then goes through additional convolutional ⁠ layers before being passed to another pooling layer. This process continues until reaching the final ⁠ convolutions and pooling layer steps. Each time, the output size ⁠ decreases while maintaining depth.

#### 3.3.2 Proposed model DenseNet201

Another among the DenseNet set of architectures created for image classification is DenseNet201. This was the ImageNet challenge's 2015 top-performing model. DenseNet layers have immediate accessibility to both the color gradients of the Loss function and the initial input image. DenseNet is a great option for image classification jobs due to the greatly decreased computing cost [53]. The network loaded into pre-trained weightiness from the ImageNet database.

The architecture of DenseNet201 is illustrated in Fig. 6, with the primary element being the dense block. Similar to the residual structure in ResNet [54], a dense block is divided into two parts: the backbone and the residual edge. The backbone consists of a 1 × 1 convolution followed by a 3 × 3 convolution, both with a stride of 1 × 1, while the residual edge remains unprocessed. These two parts are then merged using a concatenation layer to integrate the features. DenseNet201 is built by stacking multiple dense blocks along with convolutional and pooling layers.

The article "Face detection based on K-medoids clustering and associated with convolutional neural networks" was retracted in 2025. Reasons: suspected computer-generated content; unreliable results or conclusions; concerns about the citations.

### 3.4 Model evaluation and verification

The confusion matrix, sometimes referred to as the error matrix, evaluates the precision of a classifier's categorization. When analyzing the output of binary regression models like logistic regression and SVM, the confusion matrix is often employed shown in Fig. 7. The accurate rate of 0-value prediction, the correct rate of 1-value prediction, and the total prediction rate in the model outputs may all be expressed quantitatively using this approach [55].

**Fig. 7:** Confusion matrix.

**Precision:** Precision is defined as the ratio of accurately anticipated positive occurrences to all expected positive outcomes.

$$\mathrm{Pr}\;ecision=\frac{TP}{TP+FP}$$

**Sensitivity:** Sensitivity is usually calculated as follows and is the only precise positive metric that is proportionate to the total number of instances:

$$Sensitivity=\frac{TP}{TP+FN}$$

Recall and “True positive rate” are two more terms for sensitivity (TPR)

**Specificity:** The concept of "specificity" refers to the quantity of accurately identified and calculated true negatives and the technique below may be used to calculate it. $Accuracy=\frac{TP+TN}{TP+FP+FN+TN}$.

$$Specificity=\frac{TN}{TN+FP}$$

**Accuracy:** The accuracy is the sum of all instances that were successfully identified across all cases. Accuracy is measurable by

$$Accuracy=\frac{TP+TN}{TP+FP+FN+TN}$$

**F1-Score:** The F1-score is the harmonic mean of recall and accuracy. The F1 score of 1, which represents perfect recall and accuracy, is the highest achievable. $F1-Score=\frac{2\times \text{Re}call\times \mathrm{Pr}\;ecision}{\text{Re}call+\mathrm{Pr}\;ecision}$.

#### 3.4.1 ROC curve

A thorough indication of response sensitivity and particular factors is the Receiver Operating Characteristic (ROC) curve [55]. The specificity of the ROC curve's X-axis, which is used to quantify the risk of landslides, represents the likelihood that non-disaster points would be incorrectly predicted. The sensitivity, which represents the probability of the crisis point being predicted correctly, is shown on the Y-axis. The size of the region bounded by the curve and the abscissa is a measure of the model's predictive power. The accuracy of the model increases with the distance of the curve from the top left corner. The range of area under the curve (AUC) values is [0, 1], and the term “area under the curve” is used. AUC values that are nearer 1 show that the model is more accurate.

### 3.5 Classification model

#### 3.5.1 Support vector machine (SVM)

In this section, we opted for Support Vector Machines (SVM) due to their outstanding capability in handling problems that are not linearly separable. SVM can identify an optimal separating hyperplane that maximizes the margin between training samples. The objective of SVM is to minimize empirical risk and confidence interval, thereby achieving robust statistical rules for samples and enhancing the generalization capability of machine learning models. For problems that are not linearly separable, SVM projects input data from a low-dimensional space into a high-dimensional feature space, facilitating easier separation.

The article "Face detection based on K-medoids clustering and associated with convolutional neural networks" was retracted in 2025. Reasons: suspected computer-generated content; unreliable results or conclusions; concerns about the citations.

The element of face detection picture deformation is simulated using Deep neural networks like VGG-16, VGG-19, and ReseNet201, and then identified using SVM. CNN typically makes use of the SoftMax classifier. Assuming that the weight of the one before the last layer to the SoftMax layer and its activation value are the same, the SoftMax layer's input may be interpreted as following Eq. (8).

(8) $$a_{i}=\sum_{k}h_{k}w_{k}$$

Consider the following for this N-class classification method: let N be the number of nodes in the SoftMax layer and every node is registered as $p_{i}$, where i = 1,2, ….N, and $p_{i}$ is a discrete probability distribution such that $\sum_{i=1}^{N}p_{i}=1$. Among them

(9) $$p_{i}=\frac{\exp\left(a_{i}\right)}{\sum_{j=1}^{N}a_{j}}$$

The solution to equation (9) is used to compute the cross-entropy loss function of SoftMax. CNNs can gather visual data short of delivering the best categorization results. SVM with a fixed kernel function is unable to learn the complex image properties. The “soft interval” method may be used to increase the interval to gain any determining planes. Thus, the classification problem may be best resolved in the learning feature space. SVM is commonly used in data analysis, pattern recognition, regression analysis, and other fields including supervised machine learning. Standard SVM predicts which of the two categories each input belongs to, making it a non-probabilistic binary linear classifier. The following is the fundamental tenet of SVM [56].

Setup the training set data samples as follows: $\left\{\left(x_{i},y_{i}\right)|x_{i}\in R^{d},y_{i}\in \left\{-1,1\right\},i=1,2,\ldots ,N\right\},y_{i}$ for the category name d for the data's dimension and N for the training datasets. There is a generalized optimum categorization hyperplane for linearly separable data sets:

(10) w.x+b=0

Eq. (10) elements work in concert to provide the class interval with the best result, with $\frac{1}{2}{\left\|w\right\|}^{2}$ the lowest and $\frac{2}{\left\|w\right\|}$ the highest. Among these, b is an offset, dot is an inner product operator, and w is an n-dimensional vector. As a result, the following categories may be added to the optimizing problem categorization as shown in Eq. (11).

(11) $$\min\frac{1}{2}{\left\|w\right\|}^{2}\;\text{such}\;\text{that}\;y_{i}\left(w^{T}x_{i}+b\right)\geq 1,i=1,2,\ldots ,n\;i=1,2,\ldots ,n$$

The learning method used by CNN minimizes errors in the training samples by using empirical risk reduction. Once the backpropagation approach has identified the first classification hyperplane, the training procedure concludes, regardless of whether it is a local or global maximum. The most useful method for classifying SVM on a global scale is using the structure-based risk-reduction principle. SVM provides superior generalization capabilities compared to multi-layered neural networks. Replacing CNNs SoftMax layer with SVM will enhance the classification performance.

The article "Face detection based on K-medoids clustering and associated with convolutional neural networks" was retracted in 2025. Reasons: suspected computer-generated content; unreliable results or conclusions; concerns about the citations.

## 4 Results and discussions

We used the MATLAB program to implement the above-mentioned approaches. All tests utilize a Lenovo machine with an Intel(R) Core (TM) i5-1021U CPU running at 2.11 GHz. It meets the following requirements: 512 GB Solid-state Drive and 8.00 GB Random Access Memory (RAM) used for the training process. The dataset was used for training 90 % and testing 10 % during the training process. Execution time has taken around 3–4 h for 30 epochs, furthermore, we can achieve dynamic performance for the proposed model with high-end processors. The primary goal of evaluate the K-means, K-medods, and FKM clustering methods on the dataset for segmentation before giving it to the CNN architecture. This study evaluated to classify Face mask classification using deep CNN, which is more accurate than current state-of-the-art methods. The next subsections go through the operation of the categorization model. The output results for our suggested approaches utilizing pre-trained models. For this research, three different pre-trained architectures (VGG-16, VGG-19, and DenseNet201) are used, with SVM for the classification of face mask detection.

In the second experimental configuration, a completely linked layer with 10 neurons replaces the previous fully connected layer, which had 1000 neurons. The face image dataset, which contains two classes(with mask and without mask), was utilized to train all three pre-trained models that are being analyzed here. As a result, the final layer includes 1000 neurons.

### 4.1 Results of K-means clustering with pre-trained models

Mask detection techniques may assist with pre-processing with K-means clustering. It could be possible to identify possible face regions for further mask detection processing by segmenting the image into areas depending on intensity. This will be helpful for images with distracting backdrops or different lighting conditions. This paper provides our first findings for the image pre-processing applied to the face image dataset before giving it to CNN. The K-means clustering used for the face mask images will reduce the noise data. This method of clustering selects the usual of connected data points. The K value represents the cluster of centroids. Where K = 4 to initialize the face image dataset is used.

The article "Face detection based on K-medoids clustering and associated with convolutional neural networks" was retracted in 2025. Reasons: suspected computer-generated content; unreliable results or conclusions; concerns about the citations.

The CNN pre-trained models applied the face mask detection after the pre-processing. Although the performance of the resulting classification appears to be good, several restrictions prohibit the findings from being used more widely. To evaluate the models first selected for the binary classification task, then examined images of faces with mask and without mask. The findings were summarised in Table 4 which also included the F1-score, recall, precision, accuracy, specificity, and AUC. The highest accuracy is achieved by DenseNet201 (96.6 %) as shown in Table 3. In this part, comparison Table 4 existed for the classification performance of our three cutting-edge deep CNN models. This experiment compares the performance of the three pre-trained models for face mask identification.

**Table 3:** Performance of the k means clustering with DenseNet201.

Name	Classes		Macro AVG	Micro AVG
True positive	511	474	492.5	492.5
False positive	19	16	17.5	17.5
False Negative	16	19	17.5	17.5
True Negative	474	511	492.5	492.5
Precision	0.96415	0.96735	0.96575	0.96569
Sensitivity	0.96964	0.96146	0.96555	0.96569
Specificity	0.96146	0.96964	0.96555	0.96569
Accuracy	0.96569	0.96569	0.96569	0.96569
F-measure	0.96689	0.96439	0.96564	
Loss	0.0451			
AUC	0.9948

**Table 4:** Comparative of deep learning models.

	Model name	Precision%	Recall%	F1-Score%	Accuracy%
K-mean clustering	DenseNet201	96.97 %	97.1 %	97 %	96.7 %
	VGG16	93.5 %	93.9 %	93.6 %	93.6 %
	VGG19	94.5 %	94.8 %	94.6 %	94.5 %

Table 4 presents the DenseNet201 model surpassed the other three models by obtaining 96.7 % accuracy for face mask identification, according to these data. With a second-best accuracy of 94.5 % the VGG-19 model performed well. As opposed to VGG-16, had the lowest accuracy of all models at 93.6 %. DenseNet201 on the other hand, fared better than other models in terms of true positive rate, obtaining a recall of 97.1 %. Also interesting is the fact that our suggested Densenet201 technique achieved the best 96.7 % accuracy,97.1 % recall, 96.9 % precision, and 97 % F1 score.

Table 4 compares the accuracy, precision, recall, and F1-Score performance of a DenseNet201 the most accurate model. Consequently, the DenseNet201 model outperforms all other challenging methods based on different backbones. Fig. 8 represents the confusion matrices for binary classification(with mask and without mask) performance of the DenseNet201, VGG16, and VGG19 models. Fig. 8 shows the confusion matrix of the pre-trained models when applied to the face dataset. It can be observed that the proposed model DenseNet201(96.6 %) achieved high accuracy. The lowest accuracy is achieved by VGG -16(93.5 %).

The article "Face detection based on K-medoids clustering and associated with convolutional neural networks" was retracted in 2025. Reasons: suspected computer-generated content; unreliable results or conclusions; concerns about the citations.

**Fig. 8:** (a–c) Represents the Depicts of the confusion matrices of with mask and without mask images.

Our work focused on our three recognized pre-trained CNN models; these algorithms should provide a probability to each picture that shows in what way prospective it is to be classified as a face mask. By comparing these probabilities to a beginning, it is possible to create a binary label indicating the with and without face mask. Fig. 9 displays the with-mask and without a mask using this probability distribution, all with-mask samples should have a projected probability close to 1. In terms of prediction probability, DenseNet201 beat all other models.

**Fig. 9:** (a–c) Illustrates the graphics that depict the expected probability scores of both mask- and non-mask images.

To provide a summary of the results of each of these techniques, this work has included ROC curves. It performed an investigative investigation to evaluate the performance of various methods in terms of a probability model's histogram, ROC and AUC curves, precision-recall curve, accuracy, sensitivity, specificity, and F1 score. The suggested method performs better for classifying with-mask and without-mask detection than the current approaches. Fig. 10 presents the precision-recall and ROC curves for the test set, showcasing the performance of each of the three pre-trained models. DenseNet201 achieves the highest precision(96.97 %) and recall (97.1 %). The pre-trained models ROC and AUC values are plotted against the test set's true positive rate (TPR) and false positive rate (FPR).

**Fig. 10:** (a–b) Represents the ROC Curve and Precision-recall curve.

**Fig. 11:** (a–b) Represents the K-medoids clustering images.

The FPR vs. TPR graphic results in the ROC curve. This demonstrates that the three model's ROC curves exhibit comparable behavior. DenseNet201 (AUC = 0.9948) exhibits the greatest performance.

### 4.2 Results of the proposed method of K-medoid clustering

K-Medoid is a point in the cluster from which dissimilarities with all the other points in the clusters are minimal. Instead of centroids as reference points in K-means algorithms, the K-medoids algorithm takes a medoid as a reference point. The details information on K-medoids is described in Section 3.

The article "Face detection based on K-medoids clustering and associated with convolutional neural networks" was retracted in 2025. Reasons: suspected computer-generated content; unreliable results or conclusions; concerns about the citations.

K-medoids is an unsupervised clustering approach where “methods” data points function as the cluster's center. A method is the cluster point with the smallest sum of distance (also known as dissimilarity) to all other cluster objects. The distance may be calculated using the Euclidian distance, the Distance measure, or any other appropriate distance function. Hence, this method separates the data into K clusters by selecting K-medoids from the sample data. Using this method approach, the K value indicates the number of clusters that need to develop. For face area segmentation, the grayscale face image is passed to the K-medoids clustering method once K = 4 has been initialized. An example of a K-medoids clustered image is shown in Fig. 11.

#### 4.2.1 Results of K-medoid clustering with pre-trained models

This section, explains about to verify the K-medoids method. Extensive pre-processing is conducted on the face mask (with and without mask) dataset. To improve classification accuracy, this study develops a collection model that combines CNN and SVM. The tests to classify with and without a mask verify the approach's influence on classification. The proposed model performs better. Evaluations have been done for the performance of the DenseNet201 model to that of various current models for this purpose. i.e.; Vgg16, and VGG-19. To assess the efficacy of the pre-trained models were selected for classification, and then evaluated face images with and without masks. The results are summarised in Table 5 which also includes the F1-score, precision, recall, specificity, accuracy, and AUC. With an accuracy of 97.7 %, DenseNet201 gives the best results. In this part, as shown in Table 6, later the comparison of the classification performance of our three cutting-edge deep CNN models was given.

**Table 5:** Performance of the K-medoid clustering with DenseNet201.

Name	Classes		MacroAVG	MicroAVG
True positive	514	483	498.5	498.5
False positive	10	13	11.5	11.5
False-negative	13	10	11.5	11.5
True negative	483	514	498.5	498.5
precision	0.98092	0.97379	0.97735	0.97745
Sensitivity	0.97533	0.97972	0.97752	0.97745
Specificity	0.97972	0.97533	0.97752	0.97745
Accuracy	0.97745	0.97745	0.97745	0.97745
F- Measure	0.97812	0.97674	0.97743	0.97745
Loss	0.0284			
AUC	0.9980

**Table 6:** Comparative of deep learning models.

	Model name	precision%	Recall%	F1-Score %	Accuracy%
K-medoids clustering	DenseNet201	98 %	97.9 %	97.9 %	97.7 %
	VGG-16	95.4 %	95.1 %	95.2 %	94.8 %
	VGG-19	97.4 %	97.7 %	97.5 %	96.2 %

This experiment compares the DenseNet201 model's face mask detection effectiveness against that of other deep learning models currently in use. The results are shown in Table 6. These results influenced us that the DenseNet201, VGG-16, and VGG-19 models were used for face mask identification. The DenseNet201 model achieved the best accuracy of 97.7 %. The least accurate model was VGG-16 which had a 96.5 % accuracy. By reaching a recall of 97.9 %, DenseNet201, on the other hand, performed well better in terms of true positive rate than other models. It should be highlighted that the four-comparator model's accuracy, which was more than 94 %, was VGG16, and VGG19. Another significant achievement was the greatest 97.7 %, precision, recall, F1 score, and accuracy for our recommended model.

The article "Face detection based on K-medoids clustering and associated with convolutional neural networks" was retracted in 2025. Reasons: suspected computer-generated content; unreliable results or conclusions; concerns about the citations.

Fig. 12 shows the confusion matrices for binary classification for the DenseNet201, VGG16, and VGG19 models. Fig. 7 shows the confusion matrix performance based on the two different classes. It classifies the face mask detection based on the TP and TN for each class, where TP means the model has detected the class correctly, while TN means the model has detected the class incorrectly. Based on the confusion matrix Densenet201(97.7 %) achieved the best accuracy compared to the other models as shown in Fig. 12. The second highest accuracy was VGG-19(96.2 %) and the lowest accuracy was VGG16 (94.8 %).

**Fig. 12:** (a–c) Represents the confusion matrices of with-mask and without-mask images.

This work focused happening our three recognized pre-trained CNN models, these algorithms should assign a probability to every picture that demonstrates how likely it is to be classified as a face mask. Compared to these probabilities with a threshold, a binary label representing whether or not the picture is of a face mask may generated. Fig. 13 shows the probability. All with-mask samples should have a predicted probability near 1, with this probability distribution, it is easy to classify a with mask and without a mask. In terms of prediction probability, DenseNet201 was superior to all other models.

**Fig. 13:** (a–c) Illustrates the predicted probability scores of images with masks and without masks.

ROC curves have been included to summarise the findings of each of these methods. Also, this work carried out an exploratory analysis of the performance of several techniques in terms of sensitivity, precision, specificity, F1-score accuracy, ROC and AUC curve, precision-recall, and a probability model's histogram. For categorizing the with-mask and without-mask detection, the suggested techniques outperform the present methods. Fig. 14 shows, for the three CNN models, the precision-recall curves for the test set. Fig. 14 displays the ROC curves with mask and without mask detection, along with the test set's TPR and FPR on the vertical and horizontal axes, respectively. The three pre-trained model's performance using the ROC curve is shown in Fig. 14. The proposed model shows high performance with an AUC value of 0.9980. the model also achieves a precision of 98 % and a recall of 97.9 %.

The article "Face detection based on K-medoids clustering and associated with convolutional neural networks" was retracted in 2025. Reasons: suspected computer-generated content; unreliable results or conclusions; concerns about the citations.

**Fig. 14:** (a–b) Represents the ROC Curve and Precision-recall curve.

### 4.3 Results of fuzzy K-means clustering with pre-trained models

Fuzzy K-means clustering is an effective method for facial mask dataset analysis. It addresses the inherent ambiguity in mask data, where classification can be challenging due to elements like partial occlusions and light. This method can be used for the pre-processing of the face mask dataset. This method can remove the noise data as well as it will improve the accuracy level. The algorithm assigns partial memberships (between 0 and 1) to each data point (face image) across a predefined number of clusters (K). Using the FKM clustering approach, the K value indicates the number of clusters that need to be developed. The grayscale image is passed to the FKM clustering method for face area segmentation. It has used k = 4 clusters that have been initialized.

This work creates a combined model using CNN pre-trained models and SVM to increase classification accuracy. The tests to classify with and without a mask verify the approach's effects on classification. Evaluations have been done for the performance of the DenseNet201 model to that of various current models for this purpose i.e.; Vgg16, and VGG-19. To assess the efficacy of the pre-trained models were selected for classification, and then evaluated face images with and without masks. The findings are summarised in Table 7 with the F1-score, precision, recall, specificity, accuracy, and AUC. The most accurate algorithm is DenseNet201, which achieves 97.3 % accuracy.

**Table 7:** Performance of the fuzzy k- means clustering with DenseNet201.

Name	Classes		MacroAVG	MicroAVG
True positive	510	483	496.5	496.5
False positive	10	17	13.5	13.5
False-negative	17	10	13.5	13.5
True negative	483	510	496.5	496.5
precision	0.98077	0.966	0.97338	0.97353
Sensitivity	0.96774	0.97972	0.97373	0.97353
Specificity	0.97972	0.96774	0.97373	0.97353
Accuracy	0.97353	0.97353	0.97353	0.97353
F -measure	0.97421	0.97281	0.97351	0.97353
Loss	0.0304			
AUC	0.9980			

This experiment compares the DenseNet201 model's face mask detection effectiveness against that of other deep learning models currently in use.

Table 8 represents the results of data discovered that the DenseNet201 model beat the other three models for face mask recognition, obtaining 97.3 % accuracy. VGG-19 obtained the second-highest accuracy of 96 % Among all models, VGG-16 had the lowest accuracy of 95.3 %. DenseNet201, on the other hand, beat other models in terms of true positive rate, with a recall of 96.7 %. Fig. 15 represents the confusion matrices for binary classification for the DenseNet201, VGG-16, and VGG-19 models. Each confusion matrix represents the accuracy of each model. Fig. 15 shows the Densenet201(97.3 %) achieved the highest accuracy.

The article "Face detection based on K-medoids clustering and associated with convolutional neural networks" was retracted in 2025. Reasons: suspected computer-generated content; unreliable results or conclusions; concerns about the citations.

**Table 8:** Comparative of deep learning models.

	Model Name	Precision %	Recall %	F1-Score%	Accuracy %
Fuzzy k-Means	DenseNet201	98 %	96.7 %	97.3 %	97.3 %
	VGG-19	96.2 %	96.2 %	96.2 %	96 %
	VGG-16	95.6 %	96 %	95.8 %	95.3 %

**Fig. 15:** (a–c) Represents the confusion matrices of with-mask and without-mask images.

This research mainly focused on their popular, already-trained CNN models. These algorithms should assign a probability to every picture that demonstrates how likely it is to be classified as a face mask. Comparing these probabilities to a threshold can result in a label with a binary value that indicates the probability that the image depicts a face mask. Fig. 16 shows the probability. All with-mask samples should have a predicted probability near 1, with this probability distribution, it is easy to classify a with mask and without a mask. In terms of prediction probability, DenseNet201 was superior to all other models.

**Fig. 16:** (a–c) the predicted probability Scores of with-mask and without-mask images.

ROC curves are included to summarise the findings of each of these models. The exploratory analysis of a probability model's performance using several approaches, looking at its precision, sensitivity, specificity, F1-score, accuracy, ROC and AUC curve, precision-recall curve, and histogram has been done. For categorizing the with-mask and without-mask detection, the suggested techniques outperform the present methods. Fig. 17 displays the test set precision-recall curves for each of the three CNN models. The TPR and FPR of the test set are shown on the vertical and horizontal axes, respectively, in Fig. 17, which also displays ROC and AUC measures.

**Fig. 17:** (a–b) Represents the ROC Curve and Precision-recall curve.

By graphing the FPR vs. the TPR, the ROC curve is created. It can be seen from this that the three model's ROC curves exhibit similar behavior. DenseNet201 (AUC = 0.9980) shows the greatest performance.

### 4.4 Comparative scheme

Compared to the current methods such as K-means clustering, K-medoids, and FKM clustering for image pre-processing with our techniques. It was observed that as the noise density ⁠ increases, the performance of clustering algorithms decreases. Furthermore, the effects of salt and pepper noise and Gaussian noise on clustering outcomes are comparable.⁠

Table 9 shows the comparison between different pre-processing approaches on CNN pre-trained models. Our proposed method with the pre-trained model DenseNet201 achieves an accuracy of 97.7 %, precision of 98 %, recall of 97.9 %, and F1-Score of 97.9 %, the best results for face identification. Although VGG 16 and VGG19 have comparable accuracy, both models are difficult because of their huge number of parameters. The K-medoids cluster pre-processing of the face dataset with CNN pre-trained model DenseNet201 achieved the highest accuracy of 97.7 %, precision of 98 %, recall of 97.9 %, and F1-Score of 97.9 %. CNN of different models developed to simulate various data clustering combinations used for training and testing datasets. The emphasized values represent the greatest degree of performance.

The article "Face detection based on K-medoids clustering and associated with convolutional neural networks" was retracted in 2025. Reasons: suspected computer-generated content; unreliable results or conclusions; concerns about the citations.

**Table 9:** Comparative of the Semisupervised learning methods with pre-trained models.

	Model	Precision%	Recall%	F1-Score	Accuracy%
K-means Clustering	**DenseNet201**	**96.97 %**	**97.1 %**	**97 %**	**96.7 %**
	VGG16	93.5 %	93.9 %	93.6 %	93.6 %
	VGG19	94.5 %	94.8 %	94.6 %	94.5 %
K- medoids	**DenseNet201**	**98 %**	**97.9 %**	**97.9 %**	**97.7 %**
	VGG16	95.4 %	95.1 %	95.2 %	94.8 %
	VGG19	97.4 %	97.7 %	97.5 %	96.2 %
Fuzzy K-means clustering	**DenseNet201**	**98 %**	**96.7 %**	**97.3 %**	**97.3 %**
	VGG16	95.6 %	96 %	95.8 %	95.3 %
	VGG19	96.2 %	96.2 %	96.2 %	96 %
Without pre-processing	**DenseNet201**	**79 %**	**78 %**	**78 %**	**80 %**
	VGG16	75 %	74.3 %	74.2 %	75 %
	VGG 19	**72.3 %**	**73 %**	**73 %**	**72.5 %**

The pre-processing of various models on the approached K-medoids clustering, K-means, FKM, and without segmentation has been updated in Table 8. This work projected that the model with pre-trained DenseNet201 shows an accuracy of 97.7 %, an F1 score of 97.9 %, a precision of 98 %, and a Recall of 97.9 %. The segmentation of the dataset has been used for three clustered methods: K-means, FKM, and K-medoids. K-medoids have done the best segmentation on the face dataset trained with a CNN-pre-trained model, and DenseNet201 achieved the best accuracy of 97 % and 98.3 %. In our proposed K-medoids clustering using the dataset samples, the approach of substituting out the sample with and without a mask has been done. At last, the categorization of dataset samples has confirmed the adaptability of our model. Our proposed method with DenseNet 201 achieves the best accuracy compared to the other models as shown in Table 10.

**Table 10:** Comparison with existing state-of-art methods.

Author	Method	Accuracy
Lakshmi and Das 2023 [57]	K means clustering with CNN pre-trained models (DenseNet201, VGG-19, VGG-16, ResNet101, ResNet50, and AlexNet) with SVM	92.25 %
Umer et al., 2023 [31]	Depth-wise separable convolutional neural networks	94.1 %
Dash, Sethy, and Behera 2023 [43]	Pre-trained Convolutional Neural Networks	96.5 %
Balasubaramanian et al., 2023 [42]	Histogram normalization with RCNN	96 %
**Proposed method**	**K medoid clustering with CNN pre-trained models VGG16, VGG 19, and DenseNet201with SVM**	**97.7 %**

In the case of the dataset, there are only two classes (with mask and without mask), this additionally proposed a K-medoids clustering model which gives the best result with the pre-trained model DenseNet201 among all models. Then, for the classification of these two different classes, our proposed method explains the K-medoids of our DenseNet201 model, which has an accuracy of 97.7 %, a precision of 98 %, and a recall of 97.9 %. When used on the test set of the pre-trained models, the proposed method's confusion matrix is shown in Fig. 12. The model has a very high degree of accuracy while making predictions without the use of a mask. A mask results in the highest accuracy DenseNet201 achieved 97.7 % and 97.9 % recall.

The article "Face detection based on K-medoids clustering and associated with convolutional neural networks" was retracted in 2025. Reasons: suspected computer-generated content; unreliable results or conclusions; concerns about the citations.

The proposed model can utilize different types of applications such as medical image segmentation in real-time, such as distinguishing between different tissue types in MRI or CT scans. This aids radiologists in quickly identifying regions of interest. This method will aim to identify face masks from live streaming in crowded areas as well and assess, if Densenet201 may assist for better results.

The limitations of the method are representing each cluster center, the K-medoids algorithm chooses a single actual data point from a given dataset. The K-medoid method thus offers a more accurate assessment of the cluster centers. When applying the K-medoids clustering approach, the K value denotes the number of clusters that must develop. The grayscale face picture is sent to the K-medoids clustering method designed for face surface segmentation once K = 4 has been initialized. As the cluster centers expand, faces acquire more complex geometric and textural characteristics that could deviate from the algorithm's assumption of simple spherical clusters due to some drawbacks. As a result, this disparity may result in less accurate categorization and less-than-ideal cluster placements.

## 5 Conclusion

In this research, deep CNN pre-trained models VGG16, VGG19, and DenseNet201 are utilized to categorize face detection with mask and without mask. Additionally, K-means, K-medoids, and FKM clustering are used for the pre-processing of the dataset. Our proposed model K-medoids for pr-processing with DenseNet201 achieves a high 97.7 % Accuracy. However, the accuracy of the proposed method worked, and among our three pre-trained models, the best result was DenseNet201 with 97.7 % after pre-processing of the dataset. Although the model used in this research performs comparably to those without pre-processing, K-means, and FKM approaches, the result shows that the K-medoids with the DenseNet201+SVM model are well-trained. Additionally, the effectiveness of the suggested method gave the best results for images after segmentation of the dataset DenseNet201 giving the best accuracy.

The article "Face detection based on K-medoids clustering and associated with convolutional neural networks" was retracted in 2025. Reasons: suspected computer-generated content; unreliable results or conclusions; concerns about the citations.

The K-medoid clustering method has shown superior performance compared to the traditional K-means and FKM clustering methods for the pre-processing of the dataset. The experimental findings demonstrate that the K-medoid clustering technique can be used as an image segmentation tool for image processing in face masks. Moreover, there is a need to enhance the segmentation efficiency of K-medoids to fulfill the requirements of real-time applications. The next research will prioritize and examine the segmentation efficiency of K-medoids.

This demonstrates that the proposed combination of Densenet201+ SVM architecture is the most effective among those considered and is also suitable for demonstrating real-time capabilities. The real-time limitations are very beneficial for an image and video processing application including these. One additional contribution of this research is to demonstrate the advantages of the proposed Densenet201+SVM model compared to other comparable models utilized for face mask identification activities.

## Data availability

The datasets generated and analyzed during this study are available at https://www.kaggle.com/datasets/ashishjangra27/face-mask-12k-images-dataset.

## CRediT authorship contribution statement

**Potharla Ramadevi:** Writing – review & editing, Writing – original draft, Validation, Methodology, Investigation, Formal analysis, Data curation. **Raja Das:** Visualization, Supervision, Conceptualization.

## Declaration of competing interest

The authors declare that they have no known competing financial interests or personal relationships that could have appeared to influence the work reported in this paper.

## References

[1] Suryawanshi Y., Meshram V., Meshram V., Patil K., Chumchu P. (Dec. 2023). Face mask wearing image dataset: a comprehensive benchmark for image-based face mask detection models. Data Br.

[2] Manohar B., Das R. (Aug. 2023). Comparison of hybrid artificial neural networks with GA, PSO, and RSA in predicting COVID-19 cases: a case study of India. Multi-Disciplinary Appl. Fog Comput. Responsiveness Real-Time.

The article "Face detection based on K-medoids clustering and associated with convolutional neural networks" was retracted in 2025. Reasons: suspected computer-generated content; unreliable results or conclusions; concerns about the citations.

[3] Leung N.H.L. (May 2020). Respiratory virus shedding in exhaled breath and efficacy of FaceMasks. Nat. Med..

[4] Manohar B., Das R. (Jun. 2023). Artificial neural networks for prediction of COVID-19 in India by using backpropagation. Expert Syst..

[5] Feng S., Shen C., Xia N., Song W., Fan M., Cowling B.J. (May 2020). Rational use of face masks in the COVID-19 pandemic. Lancet Respir. Med..

[6] Zafeiriou S., Zhang C., Zhang Z. (2015). “Accepted manuscript A survey on face detection in the wild: past, present and future. CVIU.

[7] Kumar A., Kaur A., Kumar M. (Aug. 2019). Face detection techniques: a review. Artif. Intell. Rev..

[8] Alrammahi A.H.I., Radif M.J. (Oct. 2019). Neural networks in business applications. J. Phys. Conf. Ser..

[9] Chen Y., Wu L., Wang G., He H., Weng G., Chen H. (Sep. 2023). An active contour model for image segmentation using morphology and nonlinear Poisson's equation. Optik.

[10] Pratondo A., Chui C.K., Ong S.H. (Feb. 2017). Integrating machine learning with region-based active contour models in medical image segmentation. J. Vis. Commun. Image Represent..

[11] Li H., He H., Wen Y. (2015). Dynamic particle swarm optimization and K-means clustering algorithm for image segmentation. Optik.

[12] Ha J., Kambe M., Pe J. (2011).

[13] Sureja N., Chawda B., Vasant A. (Jun. 2022). An improved K-medoids clustering approach based on the crow search algorithm. J. Comput. Math. Data Sci..

[14] Abbasi S., Abdi H., Ahmadi A. (Mar. 2021). Int. Comput. Soc. Iran Comput. Conf..

[15] Oztel I., Yolcu Oztel G., Akgun D. (Jan. 2023). A hybrid LBP-DCNN based feature extraction method in YOLO: an application for masked face and social distance detection. Multimed. Tools Appl..

[16] Mostafa S.A. (2024). A YOLO-based deep learning model for Real-Time face mask detection via drone surveillance in public spaces. Inf. Sci..

[17] Bouhsissin S., Sael N., Benabbou F. (2021). Proc. - 2021 Int. Conf. Digit. Age Technol. Adv. Sustain. Dev. ICDATA 2021.

[18] Dash A., Sethy P.K., Behera S.K. (2023). Maize disease identification based on optimized support vector machine using deep feature of DenseNet201. J. Agric. Food Res..

[19] Simonyan K., Zisserman A. (Sep. 2014). 3rd Int. Conf. Learn. Represent. ICLR 2015 - Conf. Track Proc..

[20] Guo S., Chen S., Li Y. (2017). 2016 IEEE Int. Conf. Inf. Autom. IEEE ICIA 2016.

[21] Ha J., Kambe M., Pe J. (Jan. 2011). Data mining: concepts and techniques. Data Min. Concepts Tech..

[22] Lucasius C.B., Dane A.D., Kateman G. (Oct. 1993). On k-medoid clustering of large data sets with the aid of a genetic algorithm: background, feasiblity and comparison. Anal. Chim. Acta.

The article "Face detection based on K-medoids clustering and associated with convolutional neural networks" was retracted in 2025. Reasons: suspected computer-generated content; unreliable results or conclusions; concerns about the citations.

[23] Yang T.F., Zhang X.P. (2010).

[24] Ruspini E.H. (Jul. 1969). A new approach to clustering. Inf. Control.

[25] Pal N.R., Pal K., Keller J.M., Bezdek J.C. (Aug. 2005). A possibilistic fuzzy c-means clustering algorithm. IEEE Trans. Fuzzy Syst..

[26] Zhao X., Nie F., Wang R., Li X. (2022). Improving projected fuzzy K-means clustering via robust learning. Neurocomputing.

[27] Abou Chaaya J., Zaraket B., Harb H., Mansour A. (2023).

[28] Wang G., Jo l P. (2020). Sci. Total Environ..

[29] Ejaz M.S., Islam M.R., Sifatullah M., Sarker A. (May 2019). 1st Int. Conf. Adv. Sci. Eng. Robot. Technol. 2019, ICASERT 2019.

[30] Pan Z., Jin P., Lei J., Zhang Y., Sun X., Kwong S. (Oct. 2016). Fast reference frame selection based on content similarity for low complexity HEVC encoder. J. Vis. Commun. Image Represent..

[31] Umer M. (May 2023). Face mask detection using deep convolutional neural network and multi-stage image processing. Image Vis Comput..

[32] Ho H.T., Chellappa R. (2013). Pose-invariant face recognition using Markov random fields. IEEE Trans. Image Process..

[33] Shijie J., Peiyi J., Siping H., Haibo Sl (Dec. 2017).

[34] Nieuwenhuizen A.T., Hemming J., Suh H. (2018).

[35] sheikh B.U.H., Zafar A. (2024). Beyond accuracy and precision: a robust deep learning framework to enhance the resilience of face mask detection models against adversarial attacks. Evol. Syst..

[36] haque Sheikh B.U., Zafar A. (2024). Untargeted white-box adversarial attack to break into deep learning based COVID-19 monitoring face mask detection system. Multimed. Tools Appl..

[37] Li X., Yang Z., Wu H. (2020). Face detection based on receptive field enhanced multi-task cascaded convolutional neural networks. IEEE Access.

[38] Biju A., Edison A. (Dec. 2020). 2020 IEEE Recent Adv. Intell. Comput. Syst. RAICS 2020.

[39] Mellouk W., Handouzi W. (Jan. 2020). Facial emotion recognition using deep learning: review and insights. Procedia Comput. Sci..

[40] Saravanan T.M., Karthiha K., Kavinkumar R., Gokul S., Mishra J.P. (Jan. 2022). A novel machine learning scheme for face mask detection using pretrained convolutional neural network. Mater. Today Proc..

[41] Agarwal C., Itondia P., Mishra A. (Feb. 2023). A novel DCNN-ELM hybrid framework for face mask detection. Intell. Syst. with Appl..

[42] Balasubaramanian S., Cyriac R., Roshan S., Maruthamuthu Paramasivam K., Chellanthara Jose B. (Sep. 2023). An effective stacked autoencoder based depth separable convolutional neural network model for face mask detection. Array.

[43] Dash A., Sethy P.K., Behera S.K. (Dec. 2023). Maize disease identification based on optimized support vector machine using deep feature of DenseNet201. J. Agric. Food Res..

The article "Face detection based on K-medoids clustering and associated with convolutional neural networks" was retracted in 2025. Reasons: suspected computer-generated content; unreliable results or conclusions; concerns about the citations.

[44] Rahman M.H., Jannat M.K.A., Islam M.S., Grossi G., Bursic S., Aktaruzzaman M. (Jun. 2023). Real-time face mask position recognition system based on MobileNet model. Smart Heal..

[45] Face Mask Detection ∼12K Images Dataset.” https://www.kaggle.com/datasets/ashishjangra27/face-mask-12k-images-dataset (accessed July. 7, 2024).

[46] Van der Laan M.J., Pollard K.S., Bryan J. (Aug. 2003). A new partitioning around medoids algorithm. J. Stat. Comput. Simul..

[47] kalaivani Anbarasan, “K-Medoid Clustering Algorithm-A Review.” Accessed: February. 8, 2024. [Online]. Available: https://www.academia.edu/8446443/K_Medoid_Clustering_Algorithm_A_Review.

[48] Nie F., Zhao X., Wang R., Li X., Li Z. (2022). Fuzzy K-means clustering with discriminative embedding. IEEE Trans. Knowl. Data Eng..

[49] Toğaçar M., Ergen B., Cömert Z., Özyurt F. (Aug. 2020). A deep feature learning model for pneumonia detection applying a combination of mRMR feature selection and machine learning models. IRBM.

[50] Cireşan D., Meier U., Masci J., Schmidhuber J. (Aug. 2012). Multi-column deep neural network for traffic sign classification. Neural Network..

[51] Zhang Y., Lian J., Fan M., Zheng Y. (Dec. 2018). Deep indicator for fine-grained classification of banana's ripening stages. Eurasip J. Image Video Process.

[52] Ramadevi P., Das R. (2024). An extensive analysis of machine learning techniques with hyper-parameter tuning by Bayesian optimized SVM kernel for the detection of human lung disease. IEEE Access.

[53] Amou M.A., Xia K., Kamhi S., Mouhafid M. (Mar. 2022). A novel MRI diagnosis method for brain tumor classification based on CNN and Bayesian optimization. Healthc. (Basel, Switzerland).

[54] Lakshmi M., Das R., Manohar B. (Apr. 2024). A new COVID-19 classification approach based on Bayesian optimization SVM kernel using chest X-ray datasets. Evol. Syst..

[55] Xie W., Nie W., Saffari P., Robledo L.F., Descote P.Y., Jian W. (2021). Landslide hazard assessment based on Bayesian optimization–support vector machine in Nanping City, China. Nat. Hazards.

[56] Manek A.S., Shenoy P.D., Mohan M.C., Venugopal K.R. (Mar. 2016). Aspect term extraction for sentiment analysis in large movie reviews using Gini Index feature selection method and SVM classifier. World Wide Web.

[57] Lakshmi M., Das R. (May 2023). Classification of monkeypox images using LIME-enabled investigation of deep convolutional neural network. Diagnostics.

